# Comparative Efficacy and Long-Term Outcomes of Beta-Blockers Alone or in Combination With Angiotensin-Converting Enzyme (ACE) Inhibitors in Chronic Heart Failure: A Systematic Review

**DOI:** 10.7759/cureus.74329

**Published:** 2024-11-23

**Authors:** Waleed Hassan, Shamima A Nila, Muneeb Ahmed, David O Okello, Muhammad Maqbool, Muath M Dabas, Maryam Nour, Safiyyah M Khan, Fazeela Ansari, Natasha Anum, Sheikh Pervaiz

**Affiliations:** 1 Internal Medicine, Shaikh Zayed Hospital, Lahore, PAK; 2 Internal Medicine, Cumilla Medical College Hospital, Cumilla, BGD; 3 Internal Medicine, Rawalpindi Medical University, Rawalpindi, PAK; 4 Internal Medicine, Ministry of Health, Lusaka, ZMB; 5 Internal Medicine, Shaheed Mohtarma Benazir Bhutto Medical University, Karachi, PAK; 6 Surgery, University of Jordan, Amman, JOR; 7 Family Medicine, John F. Kennedy University School of Medicine, Willemstad, CUW; 8 Emergency Medicine, Henry Ford Health System, Detroit, USA; 9 Research Methodology, California Institute of Behavioral Neurosciences and Psychology (CIBNP), Fairfield, USA; 10 Medicine and Surgery, Dubai Medical College, Dubai, ARE; 11 Internal Medicine, Liaquat University of Medical and Health Sciences, Jamshoro, PAK; 12 Internal Medicine, Nishtar Medical University, Multan, PAK

**Keywords:** ace inhibitors, beta-blockers, bisoprolol, cardiovascular mortality, carvedilol, chronic heart failure, enalapril, heart failure hospitalization, lisinopril, reduced ejection fraction

## Abstract

This systematic review provides a comprehensive comparison of beta-blockers and angiotensin-converting enzyme (ACE) inhibitors in the management of chronic heart failure (CHF), with a focus on their long-term efficacy and safety profiles. By synthesizing evidence from randomized controlled trials (RCTs) and clinical studies, the review highlights the significant benefits of both drug classes in reducing mortality and hospital readmissions, and improving patient outcomes. Beta-blockers, such as bisoprolol and carvedilol, demonstrated superior efficacy in reducing sudden cardiac death, particularly in patients with heart failure with reduced ejection fraction (HFrEF). Angiotensin-converting enzyme (ACE) inhibitors, including enalapril and lisinopril, effectively lowered overall cardiovascular mortality by targeting the renin-angiotensin-aldosterone system (RAAS) and preventing further cardiac remodeling.

The findings of this review underscore the importance of utilizing these therapies, either alone or in combination, for optimal heart failure management. Combining beta-blockers and ACE inhibitors, or integrating them with newer agents such as angiotensin receptor-neprilysin inhibitors (ARNIs) and mineralocorticoid receptor antagonists (MRAs), provides an additive benefit, improving long-term survival and reducing heart failure-related hospitalizations. The review also identifies gaps in the current literature, suggesting that future research should focus on personalized treatment approaches, longer follow-up periods, and exploring novel therapeutic combinations for diverse heart failure populations. This evidence reinforces the role of beta-blockers and ACE inhibitors as foundational therapies in CHF and offers actionable insights for clinicians to enhance patient care.

## Introduction and background

Chronic heart failure (CHF) is a complex and progressive condition that significantly impacts the lives of millions of patients worldwide. It is characterized by the heart's inability to pump sufficient blood to meet the body's metabolic demands, leading to symptoms such as dyspnea, fatigue, and fluid retention [1]. CHF is classified based on left ventricular ejection fraction (LVEF) into two main types: heart failure with reduced ejection fraction (HFrEF) and heart failure with preserved ejection fraction (HFpEF), both of which require distinct therapeutic approaches. Despite advancements in heart failure management, optimizing pharmacotherapy to improve long-term outcomes remains a clinical challenge [2].

Among the cornerstone therapies for CHF are beta-blockers and angiotensin-converting enzyme (ACE) inhibitors. Beta-blockers, such as bisoprolol and carvedilol, work by antagonizing adrenergic stimulation, thereby reducing heart rate and improving myocardial oxygen consumption [3]. ACE inhibitors, including enalapril and lisinopril, inhibit the renin-angiotensin-aldosterone system (RAAS), reducing vasoconstriction and preventing further cardiac remodeling [4]. Both drug classes have demonstrated efficacy in reducing mortality and hospitalizations in CHF patients, yet questions remain regarding their comparative long-term benefits and safety profiles.

This review is guided by the PICO (Population, Intervention, Comparison, Outcome) framework. The population includes adults with chronic heart failure, covering both HFrEF and HFpEF subtypes. The intervention being studied involves the use of beta-blockers, such as bisoprolol, carvedilol, and atenolol, while the comparison is with ACE inhibitors, including enalapril and lisinopril. The primary outcomes assessed include long-term mortality and cardiovascular hospitalizations, while secondary outcomes focus on adverse events, heart failure progression, and quality of life metrics.

The objective of this systematic review is to critically compare the efficacy and long-term outcomes of beta-blockers versus ACE inhibitors in chronic heart failure. By synthesizing evidence from the most recent clinical trials, this review provides a comprehensive overview of which therapy offers superior survival benefits, better symptom control, and improved tolerability in the context of chronic heart failure. Additionally, this review aims to identify gaps in current research, offering insights into areas that warrant further investigation. It serves as a valuable resource for clinicians making evidence-based decisions in the treatment of chronic heart failure, guiding therapy selection based on individual patient profiles and the comparative efficacy of these foundational pharmacotherapies.

## Review

Materials and methods

Search Strategy

The search strategy for this systematic review was meticulously designed following the Preferred Reporting Items for Systematic Reviews and Meta-Analyses (PRISMA) guidelines [5], aiming to identify studies that compare the efficacy and long-term outcome of beta-blockers versus ACE inhibitors in the management of chronic heart failure. A comprehensive search was performed across several major electronic databases, including PubMed, Medline, Embase, the Cochrane Library, and Scopus. The search covered studies from the inception of each database up to September 2024 to ensure a wide scope of relevant literature was captured.

A tailored combination of Medical Subject Headings (MeSH) terms and keywords was used to reflect the specific focus of our research question. These terms included “chronic heart failure”, “beta-blockers”, “ACE inhibitors”, “randomized controlled trials”, and “long-term outcomes”. Boolean operators (‘AND,’ ‘OR’) were employed to refine and enhance the search results. Example search strings included: “beta-blockers AND ACE inhibitors AND heart failure”, “chronic heart failure AND beta-blockers AND long-term outcomes”, and “ACE inhibitors AND cardiovascular mortality AND heart failure management”. Additionally, reference lists from relevant studies were reviewed to identify further eligible studies. The search also extended to trial registries and conference abstracts to capture unpublished or ongoing clinical trials. Only peer-reviewed articles published in English were included, with a focus on randomized controlled trials, cohort studies, and meta-analyses that evaluate the efficacy and safety of the interventions in patients with chronic heart failure.

Eligibility Criteria

The eligibility criteria for this systematic review were meticulously designed to focus exclusively on randomized controlled trials (RCTs) and clinical trials that compare the efficacy and long-term outcomes of beta-blockers versus ACE inhibitors in the management of chronic heart failure (CHF). Only peer-reviewed articles published in English involving adult patients diagnosed with CHF were included. The inclusion criteria specifically targeted studies evaluating key outcomes such as all-cause mortality, cardiovascular mortality, heart failure hospitalizations, and other long-term outcomes related to the effectiveness of beta-blockers and ACE inhibitors. To ensure a comprehensive and up-to-date analysis, the timeframe for inclusion extended from the inception of the databases up to September 2024.

Studies were excluded if they focused on non-comparative interventions, involved pediatric populations, or were conducted on animal models. Additionally, grey literature, such as conference proceedings, abstracts, or unpublished works, was not considered to maintain a high standard of peer-reviewed evidence. Studies that lacked sufficient detail on the intervention methods or outcome measures directly comparing beta-blockers and ACE inhibitors in CHF were also excluded. This selective approach ensures that the review remains focused on high-quality, randomized evidence, which is critical for drawing robust conclusions about the long-term efficacy of these therapies.

Data Extraction

The data extraction process for this systematic review was meticulously structured to ensure precision and reliability in gathering relevant data on the efficacy and long-term outcomes of beta-blockers versus angiotensin-converting enzyme (ACE) inhibitors in the management of chronic heart failure (CHF). Initially, two independent reviewers conducted a thorough screening of titles and abstracts to identify studies that met the inclusion criteria. Each study was classified as "relevant," "not relevant," or "possibly relevant" based on its alignment with the review’s focus. This initial screening was instrumental in narrowing down the pool of studies for full-text review.

For studies deemed potentially eligible, a full-text review was conducted, and data extraction was performed using a standardized form in Microsoft Excel. Key data points extracted included study design, sample size, interventions, outcomes, and key findings. Both reviewers independently applied the predefined eligibility criteria, and any discrepancies were resolved through discussion, with the involvement of a third reviewer when necessary. This rigorous approach ensured consistency and accuracy throughout the review process. The extracted data was organized to capture critical information such as lead author, year of publication, intervention and comparator details, study outcomes, and adverse events, ensuring a comprehensive analysis of each study in the final review.

Data Analysis and Synthesis

For this systematic review, the data analysis and synthesis were designed to qualitatively assess the efficacy and long-term outcomes of beta-blockers versus ACE inhibitors in managing chronic heart failure. Due to variability in study designs, populations, and reported outcomes, a meta-analysis was not conducted. Instead, a narrative synthesis was employed to integrate and interpret the findings from the selected RCTs and clinical trials. Key outcomes such as all-cause mortality, cardiovascular mortality, heart failure hospitalizations, and long-term functional benefits were systematically categorized and compared between beta-blockers and ACE inhibitors. This approach allowed for the identification of trends, notable differences, and common themes across the studies. The findings were synthesized to offer a comprehensive understanding of how each treatment impacted survival, hospital readmissions, and overall heart failure management, while also highlighting any adverse events associated with each drug class. The narrative synthesis provided a holistic view of the comparative effectiveness of beta-blockers and ACE inhibitors, along with identifying gaps in the current evidence and suggesting areas for future research.

Results

Study Selection Process

The study selection process followed the PRISMA guidelines, beginning with the identification of 456 records from various databases. After the removal of 78 duplicate records, 378 records were screened based on titles and abstracts. Of these, 121 were excluded for not meeting the relevance criteria. Full-text retrieval was attempted for 257 reports, but 166 were not retrieved, leaving 166 reports to be assessed for eligibility. Upon further evaluation, 79 additional reports were excluded, leading to the inclusion of 12 studies in the final review, which were considered relevant for detailed analysis. This systematic approach ensured the selection of high-quality studies that aligned with the review's focus. The study selection process is given in Figure 1.

**Figure 1:** The PRISMA flowchart represents the study selection process PRISMA: Preferred Reporting Items for Systematic Reviews and Meta-Analyses.

Characteristics of Selected Studies

The selected studies involved a diverse range of patient populations, primarily focusing on individuals with chronic heart failure (CHF), with a subset of studies targeting those with HFrEF and others with conditions such as comorbid chronic obstructive pulmonary disease (COPD) or hypertension. Interventions included beta-blockers (e.g., bisoprolol, carvedilol, and atenolol), ACE inhibitors (e.g., enalapril, lisinopril), and comprehensive pharmacological regimens combining beta-blockers, ACE inhibitors, angiotensin receptor-neprilysin inhibitors (ARNIs), and mineralocorticoid receptor antagonists (MRAs). Comparators typically involved standard therapies, such as ACE inhibitors, beta-blockers, or placebo, depending on the study. Outcomes measured were consistent across the studies, with a primary focus on mortality rates, hospital readmissions for heart failure, cardiovascular death, and treatment tolerability. The study designs were predominantly randomized controlled trials (RCTs), with some cross-trial analyses. The key findings generally underscored the efficacy of combining pharmacotherapies to improve long-term survival and reduce cardiovascular events in patients with CHF. The characteristics of the selected studies are summarized in Table 1.

**Table 1:** A summary of the characteristics of the selected studies. HFrEF: heart failure with reduced ejection fraction, ARNI: angiotensin receptor-neprilysin inhibitor, MRA: mineralocorticoid receptor antagonist, SGLT2: sodium-glucose cotransporter 2, ACE: angiotensin-converting enzyme, ARB: angiotensin receptor blocker, RCT: randomized controlled trial, HR: hazard ratio, COPD: chronic obstructive pulmonary disease, NYHA: New York heart association, NT-proBNP: N-terminal pro–B-type natriuretic peptide, GDMT: guideline-directed medical therapy, CHF: chronic heart failure, LVEF: left ventricular ejection fraction, CIBIS: cardiac insufficiency bisoprolol study, SUPPORT: supplemental benefit of an angiotensin receptor blocker in hypertensive patients with stable heart failure using olmesartan, MI: myocardial infarction, HF: heart failure, CARMEN: carvedilol ACE-Inhibitor remodeling mild CHF evaluation.

Study	Population (P)	Intervention (I)	Comparison (C)	Outcomes (O)	Study Design	Key Findings	Risk of Bias Assessment
Vaduganathan et al., 2020 [6]	Patients with chronic heart failure with reduced ejection fraction (HFrEF), age range 55-80 years	Comprehensive disease-modifying pharmacological therapy (ARNI, β-blocker, MRA, SGLT2 inhibitor)	Conventional therapy (ACE inhibitor/ARB and β-blocker)	Primary: Cardiovascular death or first hospital admission for heart failure; Secondary: Cardiovascular death, hospital admission, all-cause mortality	Cross-trial analysis of 3 RCTs (EMPHASIS-HF, PARADIGM-HF, DAPA-HF)	Comprehensive therapy reduced risk of cardiovascular death or heart failure hospitalization by 62% (HR 0.38), with additional survival benefits of 2.7 to 8.3 years, depending on age	Low risk; well-randomized with clear outcome measures, minimal attrition bias.
Kimmoun et al., 2019 [7]	900 patients admitted for acute heart failure; high risk of readmission or death within 90 days post-discharge	High-intensity care: Rapid up-titration of β-blockers, ACE inhibitors/ARBs/ARNI, and MRA to 100% of recommended doses within 2 weeks	Usual care: Discharge and management according to usual clinical practice	Primary: 90-day all-cause mortality or heart failure readmission	Multicenter, randomized, open-label, parallel-group study	The study evaluated the safety and efficacy of rapid up-titration of heart failure therapies. The high-intensity care group showed reduced readmissions and mortality compared to usual care	Some risks: open-label design introduces performance bias, but outcome assessments are reliable.
Bhatt et al., 2021 [8]	8398 patients with heart failure and reduced ejection fraction (HFrEF)	Sacubitril/valsartan	Enalapril	Primary: Use and dosing of β-blockers and MRA; Secondary: Discontinuation rates of β-blockers and MRA at 12-month follow-up	Randomized controlled trial (PARADIGM-HF)	Sacubitril/valsartan did not result in greater discontinuation or dose down-titration of β-blockers and MRA, and promoted more sustained MRA use compared to enalapril	Low risk; randomization and blinding reduce bias, clear measurement of outcomes.
Ehteshami-Afshar et al., 2021 [9]	8399 patients with heart failure with reduced ejection fraction (HFrEF), including a subset of 1080 patients with COPD (12.9%)	Sacubitril/valsartan, with background beta-blocker use where tolerated	Enalapril, with background beta-blocker use was tolerated	Primary: Hospitalizations due to heart failure, composite of cardiovascular death or heart failure hospitalization; Secondary: Cardiovascular and non-cardiovascular hospitalizations, all-cause mortality.	Randomized controlled trial (PARADIGM-HF)	COPD was associated with lower beta-blocker use (87% vs. 94%) and worse outcomes, including a 32% higher risk of heart failure hospitalization and a 17% higher risk of cardiovascular hospitalization. Sacubitril/valsartan demonstrated consistent benefits over enalapril across both COPD and non-COPD groups, reducing hospitalizations in this high-risk subgroup	Low risk; robust randomization and blinding; clear outcome reporting.
Poole-Wilson et al., 2003 [10]	3164 patients with chronic heart failure (NYHA class II-IV)	High-dose lisinopril (32.5-35 mg)	Low-dose lisinopril (2.5-5 mg)	Primary: All-cause mortality, cardiovascular mortality, sudden death, chronic heart failure death	Randomized, double-blind, parallel-group study (ATLAS)	Age, male sex, ischemic heart disease, and increased heart rate were markers for all-cause mortality. β-blockers and antiarrhythmics reduced the risk of sudden death	Low risk; double-blinding and randomization ensure minimal bias.
Fiuzat et al., 2020 [11]	838 patients with heart failure and reduced ejection fraction (HFrEF, ≤40%)	NT-proBNP−guided therapy to optimize guideline-directed medical therapy (GDMT)	Usual care	Primary: Achieving ≥50% of the target dose of β-blockers, ACE inhibitors/ARBs, or any dose of MRAs; Secondary: Hospitalizations, cardiovascular death	Randomized controlled trial (GUIDE-IT)	Only 15.5% of patients achieved optimal GDMT at 6 months, and higher doses of β-blockers and ACE inhibitors/ARBs were associated with reduced risk of HF hospitalization and cardiovascular death	Moderate risk; some attrition and potential reporting bias.
Krum et al., 2011 [12]	1010 patients with mild or moderate, stable chronic heart failure (CHF), LVEF ≤35%	Bisoprolol (β-blocker) first for 6 months, followed by a combination with enalapril	Enalapril (ACE inhibitor) first for 6 months, followed by a combination with bisoprolol	Primary: Mode of death (sudden death, pump failure death); Secondary: All-cause mortality	Randomized controlled trial (CIBIS III)	Bisoprolol-first therapy reduced sudden deaths compared to enalapril-first therapy during the first year (HR 0.54, P=0.049); however, pump failure deaths were higher in the bisoprolol group (HR 2.39, P=0.053)	Low risk; randomized, reliable reporting, clear protocol.
Sakata et al., 2015 [13]	1147 hypertensive patients with symptomatic chronic heart failure (CHF), primarily with reduced ejection fraction (HFrEF); mean age 66 years, 75% male	Addition of olmesartan to baseline therapy (ACE inhibitors and/or β-blockers)	Control (baseline therapy with ACE inhibitors and/or β-blockers)	Primary: Composite of all-cause death, non-fatal myocardial infarction (MI), non-fatal stroke, and hospitalization for worsening heart failure; Secondary: Renal dysfunction, all-cause death	Randomized, open-label, blinded endpoint study (SUPPORT Trial)	The addition of olmesartan did not improve the primary composite outcome but was associated with worsened renal function (16.8% vs. 10.7%) and increased adverse cardiac events, particularly when combined with both ACE inhibitors and β-blockers. The triple therapy group showed a higher incidence of the primary endpoint (38.1% vs. 28.2%, HR 1.47) and all-cause death (19.4% vs. 13.5%, HR 1.50), indicating potential risks associated with adding olmesartan to dual therapy	Moderate risk; open-label design may introduce performance bias.
Willenheimer et al., 2004 [14]	1000 patients with chronic heart failure (CHF)	Bisoprolol (β-blocker) monotherapy for 6 months, followed by combination therapy	Enalapril (ACE inhibitor) monotherapy for 6 months, followed by combination therapy	Primary: Combined death or hospitalization; Secondary: Tolerability of monotherapy and combination therapy	Randomized controlled trial (CIBIS-III)	The study aims to test non-inferiority of bisoprolol-first vs. enalapril-first regarding death and hospitalization, and if bisoprolol-first shows superiority, it could change the paradigm of initiating CHF therapy with β-blockers instead of ACE inhibitors	Low risk; randomization and blinding minimize bias.
Komajda et al., 2004 [15]	572 patients with mild chronic heart failure (CHF), primarily on ACE inhibitors before study initiation (65% of patients)	Carvedilol (target 25 mg bid) and/or enalapril (target 10 mg bid); carvedilol was titrated first in the combination arm	Carvedilol monotherapy vs. enalapril monotherapy	Primary: Safety and tolerability during up-titration; Secondary: Withdrawal rates, serious adverse events, all-cause mortality and hospitalization	Randomized controlled trial (CARMEN)	No significant differences in tolerability or adverse events between carvedilol and enalapril, with similar rates of withdrawal (31%, 30%, 30%) and serious adverse events (28%, 29%, 34%) in the combination, carvedilol, and enalapril arms, respectively. Mortality and hospitalization rates were also comparable. Findings suggest carvedilol and enalapril have similar tolerability profiles, challenging the perception of carvedilol’s difficult up-titration	Low risk; strong randomization, minimal attrition bias.
Funck-Brentano et al., 2011 [16]	1010 patients with stable chronic heart failure (CHF); mean age 72.4 years; mean LVEF 28.8%	Bisoprolol (target dose 10 mg o.d.) monotherapy followed by combination with enalapril	Enalapril (target dose 10 mg b.i.d.) monotherapy followed by combination with bisoprolol	Primary: Mortality or all-cause hospitalization; Secondary: Mortality, cardiovascular hospitalization	Post hoc analysis of the CIBIS III trial	The order of drug initiation affects whether CHF patients reach target doses. The monotherapy phase was a strong independent predictor of outcomes. Older age, NYHA class III, renal impairment, and low blood pressure were associated with lower doses reached	Moderate risk; post hoc analysis may introduce selection bias.
Sturm et al., 2000 [17]	100 patients with class II or III heart failure and LVEF ≤25%, pretreated with high-dose enalapril (40 mg/day)	Atenolol (β1-blocker) 50-100 mg/day	Placebo	Primary: Combined worsening heart failure or death; Secondary: Hospitalizations for cardiac events, arrhythmias	Double-blind, placebo-controlled trial	Atenolol significantly reduced worsening heart failure and cardiac event hospitalizations compared to placebo. Fewer deaths and arrhythmia-related hospitalizations were observed in the atenolol group	Low risk; well-blinded, consistent outcome measures.

Discussion

The findings of this systematic review are consistent with a large body of literature that supports the use of beta-blockers and ACE inhibitors as foundational therapies for chronic heart failure (CHF) [18]. Previous landmark studies, such as the MERIT-HF and COPERNICUS trials, have long established the mortality benefits of beta-blockers, particularly in patients with heart failure with reduced ejection fraction (HFrEF), where they have been shown to significantly reduce both sudden cardiac death and hospitalizations for heart failure [19]. Similarly, ACE inhibitors, as demonstrated in studies like the CONSENSUS and SOLVD trials, have been proven to reduce mortality and improve survival in heart failure patients by mitigating the effects of the renin-angiotensin-aldosterone system (RAAS) [20]. Our review aligns with these findings, particularly in the observed reductions in cardiovascular mortality and heart failure-related hospitalizations when beta-blockers and ACE inhibitors are used in combination. Studies such as Vaduganathan et al. reaffirm the superior efficacy of comprehensive therapy that includes both drug classes, along with newer agents such as angiotensin receptor-neprilysin inhibitors (ARNIs) and mineralocorticoid receptor antagonists (MRAs) [6].

However, this review also highlights contrasting insights when compared to more recent literature that emphasizes individualized treatment approaches based on patient profiles. For instance, our review found that beta-blockers reduced sudden cardiac death more effectively than ACE inhibitors, as demonstrated by Krum et al. [12]; however, this benefit came at the cost of increased pump failure deaths, suggesting that therapy should be tailored based on specific heart failure phenotypes. Moreover, newer therapies like sacubitril/valsartan have shown promise in improving long-term outcomes, as evidenced by Bhatt et al. [8] and Ehteshami-Afshar et al. [9], where sacubitril/valsartan promoted better sustained MRA use and reduced heart failure hospitalizations. These findings indicate a shift in the broader heart failure management landscape, where treatment strategies are becoming more personalized, incorporating newer agents alongside beta-blockers and ACE inhibitors, offering a more nuanced approach to optimizing care in CHF patients.

The clinical implications of this review underscore the critical role of both beta-blockers and ACE inhibitors in the optimal management of chronic heart failure, particularly in patients with reduced ejection fraction [21]. Beta-blockers, with their proven efficacy in reducing sudden cardiac death and heart failure-related hospitalizations, should be considered foundational in heart failure management, especially for long-term outcomes [22]. Clinicians can maximize the benefits by initiating beta-blockers early and titrating to the highest tolerable dose, as suggested by the findings in studies like Krum et al. [12]. Similarly, ACE inhibitors, by mitigating the effects of the RAAS system, offer substantial survival benefits and should be part of any heart failure regimen, particularly for reducing all-cause and cardiovascular mortality [23]. Importantly, combining both therapies, as shown in several studies, provides an additive effect, further improving patient outcomes while maintaining a favorable safety profile. The findings suggest that tailoring therapy based on patient-specific characteristics, such as the risk of sudden death or pump failure, can enhance long-term management and reduce hospital readmissions, highlighting the need for a personalized, evidence-based approach to chronic heart failure treatment.

This systematic review has several key strengths, notably the exclusive inclusion of randomized controlled trials (RCTs) and clinical trials, which provide the highest level of evidence for evaluating the efficacy and long-term outcomes of beta-blockers and ACE inhibitors in chronic heart failure. The strict adherence to PRISMA guidelines throughout the review process ensured a transparent, systematic approach to study selection, data extraction, and synthesis, further enhancing the reliability of the findings. Additionally, the comprehensive search strategy, which spanned multiple databases and included manual reference checks, allowed for a thorough capture of relevant literature, ensuring that the review reflected the most current and robust evidence available.

However, there are limitations to this review that must be acknowledged. The variability in study designs, patient populations, and treatment protocols across the included trials introduces heterogeneity, which may affect the comparability of results. Additionally, certain secondary outcomes, such as long-term mortality and quality of life metrics, were not consistently reported across studies, limiting our ability to comprehensively evaluate these important aspects of beta-blocker and ACE inhibitor use. The absence of standardized outcome reporting, especially for long-term adverse effects and patient-centred outcomes like quality of life, restricts our capacity to provide definitive conclusions on these parameters. These limitations may impact the generalizability of the findings and highlight the need for future research that employs more standardized methodologies and specifically addresses underreported outcomes, thereby enhancing the overall evidence base for chronic heart failure management.

Future research should focus on addressing several key gaps identified in this review. One important area for further investigation is the need for larger, more diverse trials that explore the long-term efficacy and safety of beta-blockers and ACE inhibitors across broader heart failure populations, particularly in those with preserved ejection fraction, as the majority of current data is focused on reduced ejection fraction [24]. Additionally, extended follow-up periods are crucial to better assess the durability of these treatments over time, especially regarding their impact on mortality, hospital readmissions, and quality of life. Research should also explore the efficacy of combining beta-blockers and ACE inhibitors with newer therapies, such as ARNIs, SGLT2 inhibitors, and MRAs, to determine the most effective combinations for improving outcomes in complex heart failure cases [25]. Finally, more studies are needed to investigate the role of personalized medicine in tailoring heart failure therapy based on individual risk factors and disease phenotypes, which could optimize treatment strategies and enhance patient outcomes.

## Conclusions

This systematic review highlights the significant benefits of both beta-blockers and angiotensin-converting enzyme (ACE) inhibitors in managing chronic heart failure (CHF), particularly in reducing mortality, lowering hospital readmissions, and improving long-term outcomes. The evidence consistently supports the use of these therapies, either alone or in combination, as fundamental components of heart failure treatment. Beta-blockers have demonstrated superior efficacy in reducing sudden cardiac death, while ACE inhibitors play a crucial role in mitigating the effects of the renin-angiotensin-aldosterone system (RAAS), ultimately reducing overall cardiovascular mortality. For healthcare professionals, the key takeaway is the importance of early initiation and optimal dosing of these medications while also considering patient-specific factors to tailor therapy. Combining beta-blockers and ACE inhibitors or using them alongside newer agents can significantly enhance patient outcomes, reinforcing their role as essential cornerstones in heart failure management.
